The article "LncRNA BLACAT1 Accelerates Non-small Cell Lung Cancer Through Up-Regulating the Activation of Sonic Hedgehog Pathway" was retracted in 2024. Reasons: original data or images not available; unreliable results or conclusions; concerns about the data; concerns about the images.

# LncRNA BLACAT1 Accelerates Non-small Cell Lung Cancer Through Up-Regulating the Activation of Sonic Hedgehog Pathway

**DOI:** 10.3389/fonc.2021.625253

**Published:** 2021-04-14

**Authors:** Jiwei Sun, Jingzhou Jia, Wuying Yuan, Shu Liu, Wei Wang, Lili Ge, Liyue Ge, Xiao-Jun Liu

**Affiliations:** ^1^Department of Thoracic Surgery, Henan Provincial Chest Hospital, Zhengzhou, China; ^2^Department of Respiratory, Huai'an Second People's Hospital and the Affiliated Huai'an Hospital of Xuzhou Medical University, Huai'an, China; ^3^Department of Oncology, Huai'an Second People's Hospital and the Affiliated Huai'an Hospital of Xuzhou Medical University, Huai'an, China; ^4^Department of Clinical Laboratory, Huai'an Second People's Hospital and the Affiliated Huai'an Hospital of Xuzhou Medical University, Huai'an, China; ^5^Outpatient Department of External Injury and Wound, Huai'an Second People's Hospital and the Affiliated Huai'an Hospital of Xuzhou Medical University, Huai'an, China

**Keywords:** lung cancer, BLACAT1, shh, Gli-1, Smo

## Abstract

Recently, increasing evidence has displayed that lncRNAs can exhibit crucial function in cancer progression, including lung cancer. LncRNA bladder cancer-associated transcript 1 (BLACAT1) is reported to participate in various cancers. The aim of our current study was to investigate the function of BLACAT1 in non-small cell lung cancer progression and study the functional pathway. Here, we reported BLACAT1 was significantly up-regulated in lung cancer tissues in comparison to the adjacent normal tissues, which suggested BLACAT1 might act as an oncogene in lung cancer. Then, A549 and PC9 cells were infected with BLACAT1 overexpression plasmid and shRNA. As shown, we proved up-regulation of BLACAT1 greatly induced the growth of non-small cell lung cancer cells. Reversely, knockdown of BLACAT1 reduced A549 and PC9 cell proliferation, migration and invasion. Sonic hedgehog (shh) signaling is able to exert a significant role in carcinogenesis, including lung cancer. Currently, we proved that up-regulation of BLACAT1 activated shh signaling pathway, *via* inducing shh, Gli-1 and Smo expression. shh pathway inhibitor GANT-61 reversed the effect of overexpression of BLACAT1 on non-small cell lung cancer. Moreover, we manifested that loss of BLACAT1 remarkably reduced the *in vivo* growth and metastasis of A549 cells *via* enhancing infiltrating CD3+ T cells. In conclusion, our research revealed a critical role of BLACAT1 in the modulation of non-small cell lung cancer *via* modulating shh pathway.

## Introduction

Lung cancer is a common cause of cancer-related death worldwide (1). Particularly, almost 1.4 million people have been diagnosed with lung cancer each year (2, 3). NSCLC accounts for about 80–85% and SCLC accounts for 15–20%, respectively (4). In recent years, although advancing progress has been made in lung cancer, the overall survival rate of lung cancer still remains unfavorable (5). Hence, a wide understanding of the possible mechanisms in non-small cell lung cancer is required.

LncRNAs are non-coding RNAs with a length over 200 nucleotides (6, 7). Increasing lncRNAs are reported to exhibit important roles in many processes, such as cell development, cell differentiation and cell apoptosis (8–10). Dysregulated lncRNAs are reported in multiple types of cancers (11–13). For instance, lncRNA UICLM can promote colorectal cancer through sponging miR-215 and regulate ZEB2 expression (14). GAS5 enhance the killing effect of NK cells in HCC *via* modulating miR-544 and RUNX3 (15). In addition, LINC00673 induces lung cancer development through sponging miR-150-5p (16). The biological mechanisms of lncRNAs in non-small cell lung cancer development remain poorly known.

BLACAT1 is firstly recognized in bladder cancer (17). BLACAT1 is correlated with the malignant types in SCLC (18). In our present research, we reported BLACAT1 was obviously increased in lung cancer. For another, shh signaling pathway has been reported to be physiologically activated during embryogenesis, including in lung development (19). shh signaling is also significantly reactivated in many tumors, such as lung cancer (20). Then, the biological effects of BLACAT1 on non-small cell lung cancer progression were assessed in our research. BLACAT1 could induce lung cancer progression through the activation of shh signaling. Hence, the findings reported in our study might potentiate the use of BLACAT1 interference as a potential strategy to repress non-small cell lung cancer development.

## Materials and Methods

### Clinical Subjects

Twenty paired lung cancer tissues and adjacent non-tumor tissues were collected from patients undergoing surgery at Huai'an Second People's Hospital and the Affiliated Huai'an Hospital of Xuzhou Medical University between 2012 and 2016. Before the operation, these patients received no local or systemic treatment. Meanwhile, 10 lung tissues from health donors were obtained. After tissue samples were harvested, they were snap frozen in liquid nitrogen, and stored at −80°C immediately. The study was approved by the Ethics Committee of Huai'an Second People's Hospital and the Affiliated Huai'an Hospital of Xuzhou Medical University. All the patients signed the informed consent.

### Cell Culture

Non-small cell lung cancer cells A549 and PC9 were obtained from the Institute of Biochemistry and Cell Biology of the Chinese Academy of Sciences. Cells were incubated in RPMI-1640 with 10% FBS, 100 U/ml penicillin, and 100 mg/ml streptomycin in humidified environment at 37°C with 5% CO_2_.

### Vector Construction and Lentiviral Transfection

The negative controls and shBLACAT1 were provided by Gene Pharma (Shanghai, China). Cells were infected with the lentivirus and harvested 48 h later to carry out further cell function experiments. To obtain the BLACAT1 stable knockdown cell line, cells were infected with LV-shBLACAT1 and LV-NC with 6 μg/ml polybrene and selected using 10 μg/ml puromycin. Then, pcDNA3.1-BLACAT1-OE plasmid and control pcDNA3.1 plasmid (Gene Pharma, Shanghai, China) were transfected into cells by using lipofectamine 3000.

### CCK-8 Assay

After cell infection, 3,000 cells were grown into a 96-well-plate. After 1d, 2d, 3d, and 4d, cells were added with CCK-8 (Dojindo Laboratories, Kumamoto, Japan) under the manufacturer's instructions. After 2 h, OD value was tested by the microplate reader (BioTek, Winooski, VT, USA).

### Colony Formation Assay

After infection, 400 cells were incubated for 14 days in a 6-well-plate. Then the medium was changed twice a week. Cells were washed twice using PBS, fixed in methanol and then stained by 0.1% crystal violet staining solution for 20 min. Afterwards, cells were observed and photographed.

### Cell Apoptosis Analysis

The apoptosis was detected using the Annexin VFITC/PI kit. Cells were inoculated into a 6-well-plate. Transfected cells were collected using trypsinization and re-suspended in 1 × binding buffer. Afterwards, Annexin V-FITC and PI staining was carried out in the dark for 15 min. Then, apoptotic cells were identified by a FACScan flow cytometer. Subsequently, the data were analyzed using CellQuest software.

### Scratch Assay

In brief, cells were seeded in 6-well-plates and incubated for a whole night. After appropriate cell attachment, culture inserts were removed. Then, cells were washed twice using PBS. Afterwards, at 0 and 24 h after scratch would formation, images were obtained using an inverted microscope.

### Transwell Assay

To evaluate cell migration and invasion ability, transwell migration and invasion assay were conducted. To conduct migration assay, the experiments were carried out the same as those in the invasion assay except for the Matrigel coating (BD Biosciences, Franklin Lakes, NJ, USA). After 24 h, we removed the filters. Cells adhering to the lower surface were fixed and then stained using 0.1% Crystal Violet. An inverted microscope (Olympus, Wuhan, China) was used to photograph five randomly selected fields in each well.

### *In situ* Hybridization

TMAs were de-paraffinized by immersion and rehydrated *via* serial ethanol followed by immersion in DEPC-treated PBS for 5 min (21). The BLACAT1 LNA custom detection probe was utilized to carry out. Then, slides were digested using 20 mg/ml proteinase K. Sections were prehybridized in 50% deionized formamide at 58°C for 60 min and hybridized at 58°C with 0.5 mg/ml DIG-labeled RNA probe. After hybridization, slides were treated with 20 mg/ml RNase A for half an hour and washed with 0.1X SSC at 58°C. Afterwards, hybridized probes were determined using alkaline phosphatase-conjugated anti-DIG antibody.

### qRT-PCR

TRIzol was employed to isolate total RNA (Takara, Dalian, China) and the resulting RNA molecules were reverse transcribed into cDNA by utilizing PrimeScript™ RT reagent kit (Takara, Dalian, China). qPCR was conducted using a Taq-Man 2 × Universal PCR Master Mix reagent on a CFX96™ Real-time PCR detection system. Then, primer sequences were displayed in Table 1.

**Table 1:** Primers for real-time PCR.

**Genes**	**Forward (5^**′**^-3^**′**^)**	**Reverse (5^**′**^-3^**′**^)**
GAPDH	GTCTCCTCTGACTTCAACAGCG	ACCACCCTGTTGCTGTAGCCAA
Shh	CCGAGCGATTTAAGGAACTCACC	AGCGTTCAACTTGTCCTTACACC
Gli1	AGCCTTCAGCAATGCCAGTGAC	GTCAGGACCATGCACTGTCTTG
Smo	TGCTCATCGTGGGAGGCTACTT	ATCTTGCTGGCAGCCTTCTCAC

### Western Blot

Equal proteins were subjected to 10% SDS-PAGE gels. PVDF membranes were used to transfer the protein. Then, the membranes were incubated with Shh, Gli1, Smo, and GAPDH antibodies (Cell Signaling Technology, Danvers, MA, USA) at 4°C for a whole night. Next day, the secondary antibody (Thermo Fisher Scientific, Sunnyvale, CA, USA, 1:2,000) was added. Afterwards, protein bands were visualized by enhanced chemiluminescence (ECL).

### Flow Cytometry Analysis of Ki-67

Ki-67 positive cells were assessed using flow cytometry. Ki-67 antibody (BD Biosciences, Franklin Lakes, NJ, USA) was used. Cells were washed twice using staining buffer. About 10^5^ cells were incubated with monoclonal antibodies for 45 min in the dark. Then, data were collected by FACS caliber (Becton Dickinson, NJ, USA).

### Confocal Microscopy

Cells were fixed using 4% paraformaldehyde and stained using the indicated primary antibodies (Abcam, Cambridge, USA) at 4°C. Then, secondary antibodies were used for 1 h. Nuclei were stained by DAPI (Beyotime, Shanghai, China) for 3 min. A Nikon A1r confocal microscope was used to obtain immunofluorescence.

### Tumor Xenograft Assay

Twelve six-week-old female BALB/C nude mice were obtained from Beijing HFK Bio-Technology. A549 cells down-regulated BLACAT1 were injected into BALB/C mice on the right back. Seven days later, the mice were examined 3 times every week for 1 month. Tumor volume was assessed based on the length and width of tumors. At last, mice were sacrificed *via* cervical dislocation after 17 days. Tumor tissues were extracted and collected for the subsequent researches. Animal protocol was approved by the Ethic Committee on Animal Experimentation of Huai'an Second People's Hospital and the Affiliated Huai'an Hospital of Xuzhou Medical University. Tumor and brain tissue samples were embedded in paraffin for HE staining and immunohistochemistry staining.

### Immunohistochemistry Analysis

Excised tumor tissues were fixed, dehydrated, paraffin-embedded, and then cut into sections. Afterwards, sections were analyzed using antibodies against CD3 (1:200, Abcam, Cambridge, USA) and Ki-67 (1:200, Abcam, Cambridge, USA) was used. Light microscopy (Olympus, Tokyo, Japan) was utilized and the image was quantified using Image-Pro Plus.

### Statistical Analysis

Statistical analysis was conducted using SPSS 18.0 and GraphPad Prism 6 software. Chi-square test was carried out to analyze the different distribution of clinical variables. *t*-test or analysis of variance (ANOVA) was carried out to evaluate the difference between different groups. *P* < 0.05 was statistically significant.

## Results

### BLACAT1 Is Significantly Elevated in Non-small Cell Lung Cancer

We collected lung tissues from healthy donors and lung cancer patients. qRT-PCR analysis displayed BLACAT1 expression in lung tissues was obviously increased in lung cancer patients compared to the healthy donors (Figure 1A). Besides, BLACAT1 expression level was up-regulated in a stage dependent manner in Figure 1B. In addition, BLACAT1 expression in tumor tissues was overexpressed in Figure 1C. Subsequently, RNA hybridization analysis revealed that BLACAT1 expression was strongly stained in three lung cancer patients randomly chosen (Figure 1D). These data indicated that BLACAT1 was increased in non-small cell lung cancer.

**Figure 1:** BLACAT1 is increased in lung cancer tissues. **(A)** BLACAT1 expression in lung tissues from healthy donors and lung cancer patients. **(B)** BLACAT1 expression level in different stages of lung cancer patients. **(C)** BLACAT1 expression in para-tumor and tumor tissues from lung cancer patients. **(D)** RNA hybridization analysis of BLACAT1 expression in para-tumor and tumor tissues from three lung cancer patients. (100×). **P < 0.01.

### Increased BLACAT1 Induces the Growth of Non-small Cell Lung Cancer

Then, to study the detailed role of BLACAT1, A549, and PC9 cells were infected with pcDNA3.1-BLACAT1-OE. In Figure 2A, we found BLACAT1 expression was significantly enhanced by pcDNA3.1-BLACAT1-OE. Flow cytometry indicated that Ki-67 positive cell ratio was increased in BLACAT1 over-expressed A549 and PC9 cells (Figure 2B). Flow cytometry analysis evidenced that cell apoptosis was not altered in BLACAT1 over-expressed A549 and PC9 cells in Figure 2C. In Figures 2D,E, transwell migration and invasion assay manifested overexpression of BLACAT1 suppressed A549 and PC9 cell migration and invasion. Wound closure of A549 and PC9 cells was triggered by the increased BLACAT1 (Figure 2F). These results implied that high expression of BLACAT1 promoted non-small cell lung cancer cell progression.

**Figure 2:** BLACAT1 enhances the progression of non-small cell lung cancer. BLACAT1 were overexpressed in A549 and PC9 cells using pcDNA3.1-BLACAT1-OE. **(A)** BLACAT1 expression level in A549 and PC9 cells. **(B)** Flow cytometry analysis of Ki-67 level in BLACAT1 over-expressed cells. **(C)** Flow cytometry analysis of BLACAT1 over-expressed cell apoptosis. **(D)** Transwell migration assay of BLACAT1 over-expressed cells. (100×). **(E)** Transwell invasion assay of BLACAT1 over-expressed cells. (100×). **(F)** Wound healing assay of BLACAT1 over-expressed cells. (100×). **P < 0.01.

### Decreased BLACAT1 Restrains the Progression of Non-small Cell Lung Cancer

Reversely, A549 and PC9 cells were infected with BLACAT1 shRNA. It was manifested that BLACAT1 expression level was greatly reduced by BLACAT1 shRNA *in vitro* in Figure 3A. In Figure 3B, Ki-67 positive cell percentage was decreased by loss of BLACAT1 in A549 and PC9 cells. CCK-8 assay implied the cell *via*bility was restrained by loss of BLACAT1 expression (Figure 3C). Then, transwell migration and invasion indicted A549 and PC9 cell migration and invasion was depressed by BLACAT1 shRNA as demonstrated in Figures 3D,E. These implied that loss of BLACAT1 restrained the progression of non-small cell lung cancer.

**Figure 3:** BLACAT1 inhibits the progression of non-small cell lung cancer. BLACAT1 were depleted in A549 and PC9 cells using shRNA transfection. **(A)** BLACAT1 expression in A549 and PC9 cells. **(B)** Flow cytometry analysis of Ki-67 level in BLACAT1 over-expressed A549 and PC9 cells. **(C)** CCK8 assay analysis of BLACAT1 depleted A549 and PC9 cells. **(D)** Transwell migration of BLACAT1 depleted A549 and PC9 cells. **(E)** Transwell invasion of BLACAT1 depleted A549 and PC9 cells. *P < 0.05; **P < 0.01.

### BLACAT1 Activates Shh Signaling Pathway

To further investigate how BLACAT1 contributed to lung cancer cell progression, the activity of shh pathway was assessed. As displayed in Figures 4A,B, western blot and qRT-PCR analysis proved that shh, Gli-1, and Smo expression was induced by BLACAT1 in A549 and PC9 cells. Moreover, confocal analysis indicated Gli-1 positive cells were increased by BLACAT1 overexpression in A549 and PC9 cells (Figure 4C). In Figure 4D, colony formation assay was carried out and we found that A549 and PC9 cell colony formation ability was increased by BLACAT1. GANT-61 acts as an inhibitor of shh signaling pathway and we proved that GANT-61 was able to reverse the increased cell colonies as shown in Figure 4D. These data suggested shh pathway was involved in lung cancer progression mediated by BLACAT1.

**Figure 4:** BLACAT1 activates shh signaling pathway. **(A)** Shh, Gli1, and Smo protein level in BLACAT1 over-expressed A549 and PC9 cells. **(B)** Shh, Gli1, and Smo mRNA level in BLACAT1 over-expressed A549 and PC9 cells. **(C)** Confocal analysis the expression level of Gli1 in A549 and PC9 cells. **(D)** Colony formation of BLACAT1 over-expressed A549 and PC9 cells treated with shh pathway inhibitor GANT-61. *P < 0.05; **P < 0.01.

### Loss of BLACAT1 Reduces *in vivo* Growth and Metastasis of Non-small Cell Lung Cancer

Furthermore, BLACAT1 was knockdown in A549 cells using BLACAT1 shRNA transfection. Cells were then injected into the BALB/c nude mice on the right back. In Figure 5A, we observed that tumor volume was remarkably reduced in BLACAT1-shRNA group time dependently. In Figure 5B, tumor weight was increased by BLACAT1-shRNA. Moreover, quantification of infiltrating CD3^+^ T cells was analyzed and CD3^+^ T cells were significantly enriched by silence of BLACAT1 (Figure 5C). Flow cytometry analysis indicated that Ki-67 positive cells were decreased by the loss of BLACAT1 (Figure 5D). Metastatic brain lesions were reduced in BLACAT1-shRNA mice group as confirmed using H&E staining in Figure 5E.

**Figure 5:** BLACAT1 deletion ameliorates the development of non-small cell lung cancer *in vivo*. BLACAT1 were knocked down in A549 cells using shRNA of BLACAT1. Transfected cells were injected into BALB/c nude mice on the right back. **(A)** Tumor size. Mice were injected with control and BLACAT1-shRNA A549 cells. **(B)** Tumor weight. **(C)** Immunohistochemical of infiltrating CD3+ T cells around tumors. Bar = 20 μM. **(D)** Immunohistochemical of Ki-67 from mice tissues. Bar = 50 μM. **(E)** Metastatic brain lesions in mice. Arrows indicate the metastasis brain lesions. *P < 0.05; **P < 0.01.

## Discussion

The significant data of our study is BLACAT1 demonstrates a crucial role in lung cancer development. We reported that BLACAT1 was significantly up-regulated in human lung cancer tissues. In addition, functional studies indicated that tumorigenic roles of BLACAT1 in promoting non-small cell lung cancer cell progression was involved in shh signaling pathway. Mechanistically, we found that BLACAT1 activated shh signaling pathway. These results indicated that BLACAT1 acted as a crucial oncogene in non-small cell lung cancer.

Many non-coding transcripts have been reported and lncRNAs have obtained increasing attention due to their various function. Many lncRNAs are abnormally expressed and they can exhibit multiple effects in cancer progression (22–24). As a newly discovered lncRNA, BLACAT1 is to be correlated with poor clinical outcomes in many cancers (25). For instance, lncRNA BLACAT1 can promote glioma cancer progression *via* activating Wnt pathway (26). BLACAT1 induces cervical cancer cell growth through activating Wnt pathway (27). In addition, BLACAT1 is increased in hepatocellular carcinoma and down-regulation of BLACAT1 suppressed cancer development through sponging hsa-miR-485-5p (28). In our work, we indicated a novel biological effect of BLACAT1 in non-small cell lung cancer.

In order to investigate the molecular mechanisms through which BLACAT1 regulated l non-small cell lung cancer, shh signaling pathway was concentrated. shh signaling pathway is reactivated in many solid tumors (19, 20). A better understanding of shh signaling can open an avenue for the treatment of various types of cancers (29). For example, abnormal shh signaling can attenuate lung cancer and enhance chemo-therapy (30). The shh signaling is activated by ligands and they can bind to Ptch. The process of shh ligand binding to Ptch reduces the inhibition of Smo and activates signal transduction through Gli transcription factor. Here, we observed that BLACAT1 significantly induce Shh, Gli1 and Smo expression level in A549 and PC9 cells. shh pathway inhibitor GANT-61 obviously reversed the effect of BLACAT1 on lung cancer growth. The detailed mechanism for lncRNA BLACAT1 in regulating Sonic Hedgehog pathway needs further investigation. We would like to focus on whether there is a target gene of BLACAT1 in lung cancer progression.

In our future study, we should figure out the reason for high BLACAT1 expression in non-small cell lung cancer. In addition, microRNAs have gained widespread attention for their role in diverse cancer, including lung cancer (31). The potential effect of BLACAT1 on its downstream molecular microRNAs is limited. LncRNAs can modulate various biological functions at transcriptional, post-transcriptional level and modulate protein activity (32–34). More researches are warranted to investigate the detailed function of BLACAT1 on non-small cell lung cancer.

In conclusion, our study displayed that BLACAT1 acts as a crucial oncogene in non-small cell lung cancer. BLACAT1 can promote non-small cell lung cancer cell growth *via* activating shh signaling. Our study suggests a strategy for targeting BLACAT1 as a potential biomarker in non-small cell lung cancer.

## Data Availability Statement

The raw data supporting the conclusions of this article will be made available by the authors, without undue reservation.

## Ethics Statement

The studies involving human participants were reviewed and approved by Huai'an Second People's Hospital and the Affiliated Huai'an Hospital of Xuzhou Medical University. The patients/participants provided their written informed consent to participate in this study. The animal study was reviewed and approved by Huai'an Second People's Hospital and the Affiliated Huai'an Hospital of Xuzhou Medical University.

## Author Contributions

X-JL designed the research and revised the manuscript. JS, JJ, and WY performed the experiments. JS drafted the manuscript. JJ and WY collected the data and did the analysis. All authors approved the final manuscript.

## Conflict of Interest

The authors declare that the research was conducted in the absence of any commercial or financial relationships that could be construed as a potential conflict of interest.
